The article "Beyond devices: preschoolers’ learning behaviors as moderators of the link between home digital resources and their digital literacy" was published in 2025. Journal: Front Psychol.

# Beyond devices: preschoolers’ learning behaviors as moderators of the link between home digital resources and their digital literacy

**DOI:** 10.3389/fpsyg.2025.1613793

**Published:** 2025-10-08

**Authors:** Young Kyung Moon

**Affiliations:** Department of Counseling, Daejeon City, Republic of Korea

**Keywords:** digital literacy, preschool children, learning behaviors, home digital resources, techno-subsystem, person-environmental interaction perspective

## Abstract

This study investigated how preschoolers’ learning behaviors moderate the relationship between home digital resources and their digital literacy. Digital literacy was conceptualized in two domains: operational digital literacy, which involve the ability to manipulate digital devices, and cultural digital literacy, which emphasize creative engagement and meaning-making. Participants included 514 preschool-aged children and their mothers in South Korea. Mothers reported on home digital resources and children’s learning behaviors, while validated scales were used to assess operational and cultural digital literacy. Moderation analyses tested whether competence motivation, attention/persistence, and learning strategy influenced the strength of the relationship between digital access and literacy outcomes. The results showed that access to home digital resources significantly predicted both operational and cultural digital literacy. For operational digital literacy, competence motivation and learning strategy strengthened the effect of digital access, suggesting that motivated and strategically engaged children gained greater technical benefits. Attention/persistence, however, did not moderate this relationship. For cultural digital literacy, competence motivation again acted as a positive moderator, indicating that motivated children engaged more deeply with symbolic and creative aspects of digital media. In contrast, learning strategy unexpectedly weakened the relationship, suggesting that children with less structured approaches benefited more from home digital exposure in this domain. These findings highlight that digital device access alone is not sufficient for literacy development. Children’s motivational and strategic dispositions shape how digital resources are translated into digital literacy development. Effective approaches to supporting early digital literacy should integrate both access to digital tools and opportunities to foster motivation, curiosity, and self-regulation in young learners.

## 1 Introduction

In today’s increasingly digital world, children are surrounded by technology from the earliest years of life. Mobile devices, digital applications, and online platforms are now woven into the fabric of children’s everyday experiences (OECD, 2021). This transformation has reshaped how young children play, communicate, and access information but has elevated the importance of digital literacy as a core developmental competence in early childhood (Neumann, 2016; Wood et al., 2016). With digital exposure beginning well before formal schooling, understanding how digital literacy develops during the preschool years has become a pressing priority for educators, researchers, and policymakers.

The article "Beyond devices: preschoolers’ learning behaviors as moderators of the link between home digital resources and their digital literacy" was published in 2025. Journal: Front Psychol.

Digital literacy in early childhood is now recognized not merely as technical skill but as a developmental construct reflecting how children engage with, interpret, and create meaning through digital media in social and cultural contexts. Drawing from Green (1998) tripartite model, it includes operational, cultural, and critical dimensions, with operational and cultural domains most salient in early childhood (Marsh, 2016; Neumann et al., 2017; Burnett and Merchant, 2018). Operational literacy involves the technical skills required to manipulate digital devices, such as tapping, swiping, launching applications, and adjusting settings (Neumann, 2016). In contrast, cultural literacy reflects children’s ability to engage with digital texts in creative and interpretive ways—such as storytelling, meaning-making, and digital collaboration. Operational literacy, often referred to as emergent digital literacy, is widely studied as the foundational form of digital literacy in early childhood, representing the basic skills young children develop that underpin later digital competencies (Neumann et al., 2017). In contrast, cultural digital literacy can be understood as a form of digital play, involving the integration of real-world experiences and digitally mediated interactions—through which children communicate with others, share experiences and knowledge, savor culture, and engage in creative expression (Arnott, 2017; Marsh, 2016). These domains are distinct yet interconnected, shaped by both environmental supports and child characteristics (Kumpulainen et al., 2020). However, the measuring cultural digital literacy in early childhood remains challenging, as existing scales often fail to capture children’s symbolic and collaborative use of digital media (Ollonen and Kangas, 2025).

The home environment plays a central role in digital literacy development. Johnson and Puplampu’s (2008) techno-subsystem theory offers a conceptual framework for understanding the home as a “digital microsystem,” embedded within a child’s broader ecological context. This model incorporates digital technologies—such as devices, internet connectivity, and media-related practices—as integral elements of the child’s microsystem. Within this framework, digital resources, such as devices and connectivity, function as structural affordances that provide opportunities for developmental engagement. Empirical findings consistently indicate that the presence and diversity of digital tools in the home are positively associated with children’s digital literacy (Cao et al., 2024). Yet access alone does not guarantee meaningful outcomes, as children benefit differently depending on their internal dispositions. In Korea, most preschoolers have daily access to smartphones or tablets (Korea Press Foundation, 2022; Kim and Lee, 2022), but notable disparities in digital literacy outcomes suggest environmental affordances alone cannot explain developmental variability.

The article "Beyond devices: preschoolers’ learning behaviors as moderators of the link between home digital resources and their digital literacy" was published in 2025. Journal: Front Psychol.

Children’s learning behaviors offer a critical lens for understanding this variability. Learning behaviors refer to a broad construct encompassing various skills and dispositions that reflect how young children engage with and respond to learning experiences (Domínguez et al., 2010; Fantuzzo et al., 2004). These behaviors are essential for promoting autonomous task engagement and enabling children to persist through cognitively demanding activities, thereby supporting effective learning outcomes (Fantuzzo et al., 2004; McDermott et al., 2012). McDermott et al. (2012) identify three core components of learning behavior: competence motivation (the intrinsic desire to master challenges), attention/persistence (the ability to focus and sustain effort), and learning strategy (the use of goal-directed approaches to learning tasks). Given that play is a central mode of learning for young children, it is reasonable to expect that their exploratory interactions with digital devices are also shaped by individual learning behaviors.

These traits influence the quality of children’s engagement in playful digital learning, where interactions are often spontaneous, creative, and emotionally engaging (Kangas et al., 2017; Marsh, 2016). Children might draw pictures on a tablet, narrate stories using digital apps, or engage in imaginative role-play with avatars or characters. Within these contexts, learning behaviors function as critical supports. Children are intrinsically motivated to explore and master tasks when their needs for autonomy, competence, and relatedness are fulfilled (Deci and Ryan, 1985). In contrast, children with lower levels of motivation or persistence may engage passively or disengage quickly, even when rich digital resources are available. These examples suggest that learning behaviors not only predict overall engagement but also shape the quality of interaction in digital play.

The article "Beyond devices: preschoolers’ learning behaviors as moderators of the link between home digital resources and their digital literacy" was published in 2025. Journal: Front Psychol.

From a person-environmental interaction perspective (Bronfenbrenner and Morris, 2006), developmental outcomes emerge from sustained interactions between person and context. Digital resources provide structural affordances, but children’s learning behaviors determine how effectively these affordances are transformed into literacy-building experiences. When dispositions align with contextual opportunities, developmental gains are maximized; when misaligned, benefits remain limited. This study focuses on how digital affordances in the home environment interact with individual differences in children’s learning behaviors. In particular, characteristics such as competence motivation, attention/persistence, learning strategy may influence the degree to which children meaningfully engage with digital resources, shaping their digital literacy development.

## 2 Purpose of the present study

In this study, we aim to investigate how preschoolers’ learning behaviors—namely competence motivation, attention/persistence, and learning strategy—moderate the relationship between home digital resources and young children’s digital literacy. Rather than treating the home digital environment as a composite construct, we focus on digital resources as a concrete and measurable structural feature of the child’s microsystem. Framed within Techno-sub system theory and person-environmental interaction perspective, these resources are understood as environmental affordances whose developmental impact is shaped by their fit with individual learning dispositions. By conceptualizing digital literacy in two domains—operational and cultural—and situating its development in the context of playful digital learning, this study seeks to provide a nuanced, ecologically grounded understanding of how digital competencies emerge through the interaction of internal and external factors in early childhood.

To address this aim, the study proposes a moderated model in which children’s learning behaviors influence the strength of the relationship between home digital resources and two domains of digital literacy: operational and cultural. The proposed research model is illustrated in Figure 1.

**Figure 1:** Research model.

Accordingly, the research question of this study is as follows: How does young children’s learning behaviors moderate the relationship between the home digital resources and their digital literacy?

## 3 Methods

### 3.1 Participants

The participants of this study comprised 514 mothers and their five-year-old children from Seoul, Gyeonggi, Daejeon, and Daegu in South Korea. To address a new research question, the current study reanalyzed previously collected data that had been used in earlier studies (Moon, 2025a,b; Moon and Shin, 2025), each of which examined individual variables in isolation. In contrast, this study employed a moderation analysis framework to explore whether preschoolers’ learning behaviors moderate the relationship between home digital resources and digital literacy. This approach extends previous work by integrating these factors into a unified interaction model grounded in the techno-subsystem perspective. The average daily duration of digital device use was 1.59 h (SD = 3.14) for children and 4.27 h (SD = 3.18) for mothers. The devices most frequently used by the children were tablets (37.7%) and smartphones (26.3%), whereas parents primarily used smartphones (82.9%) and computers (11.0%).

The article "Beyond devices: preschoolers’ learning behaviors as moderators of the link between home digital resources and their digital literacy" was published in 2025. Journal: Front Psychol.

### 3.2 Measures

Home digital resources, learning behaviors, children’s digital literacy were measured using validated scales. Each measure was selected for its theoretical grounding and prior use in early childhood research. Reliability coefficients for the present sample are reported in Table 1.

**Table 1:** Summary of instruments.

Construct	Subscale (No. of items)	Example item	Scale range	Reliability (*α*)
Home Digital Resources	9 items	“Child has access to a tablet”	Yes/No	0.70
Learning Behaviors	Competence Motivation (12)	“My child resists or fears new activities”	3-point	0.85
	Attention/Persistence (5)	“Child pays attention to what adults say”	3-point	0.72
	Learning Strategy (6)	“My child attempts tasks in ways that are not permitted”	3-point	0.72
Digital Literacy	Operational (16)	“Child can swipe the screen”	3-point	0.93
	Cultural (8)	“Child can explore digital storybooks”	3-point	0.86

#### 3.2.1 Home digital resources

Home digital resources were measured using a set of items adapted from previous studies by Ozturk and Ohi (2018) and Kumpulainen et al. (2020). Mothers reported the presence of nine types of digital devices (e.g., television, smartphone, tablet, computer, internet-enabled toys) available to their child. Responses were coded dichotomously (0 = not available, 1 = available) and summed to produce an overall index of home digital resources. This approach has been widely used in early childhood media studies to capture structural aspects of the digital environment.

#### 3.2.2 Learning behaviors

Learning behaviors were assessed using a Korean-translated version of the Preschool Learning Behaviors Scale (PLBS) originally developed by McDermott t al. (2012). The version used in this study consisted of 23 items: competence motivation (12), attention/persistence (5), and learning strategy (6). Each item was negatively worded and rated on a 3-point Likert scale (1 = mostly true, 2 = sometimes true, 3 = not true at all), with higher scores indicating greater levels of the respective learning behaviors.

The article "Beyond devices: preschoolers’ learning behaviors as moderators of the link between home digital resources and their digital literacy" was published in 2025. Journal: Front Psychol.

#### 3.2.3 Digital literacy

Digital literacy was assessed using a scale specifically developed to capture two distinct domains: operational and cultural digital literacy. The items were constructed to reflect children’s competencies in engaging with digital devices and applications, participating in digital communication, and creatively interacting with verbal, visual, and auditory content. Additional areas assessed included digital problem-solving, information seeking, and sharing behaviors, as described in previous studies (Lee and Kang, 2021; Marsh, 2016; McPake et al., 2012). Operational Digital Literacy (16 items) assessed children’s technical skills (e.g., swiping, launching applications, adjusting settings). Cultural Digital Literacy (8 items) captured interpretive and creative engagement, such as exploring digital storybooks or engaging in collaborative digital play. Mothers rated each item on a 3-point scale (1 = not at all, 2 = sometimes, 3 = always without adult assistance).

### 3.3 Research procedure

This study was conducted with the approval of the Institutional Review Board at Daejeon University (IRB No. 1040647-202208-HR-001-03). Participants were recruited through kindergartens, childcare centers, and online parenting communities located in several urban regions of South Korea, including Seoul, Gyeonggi, Daejeon, and Daegu. Survey participation was voluntary and informed consent was obtained from all participants prior to data collection. To reach a broad sample, approximately 700 mothers were initially invited via a digital survey link. For those unable to complete the online questionnaire, paper-based surveys were distributed directly through affiliated institutions. A total of 293 responses were gathered online, and 221 were collected through the paper survey format, yielding an overall response rate of approximately 73.4%. After excluding incomplete responses, the final sample consisted of 514 valid cases. Prior to beginning the survey, participants were fully informed of the study’s purpose, procedures, and confidentiality protocols. They were assured that their participation was entirely voluntary and that all responses would be kept anonymous and used solely for research purposes.

### 3.4 Data analysis

The data were analyzed using IBM SPSS Statistics version 26.0 and the PROCESS macro version 4.2 (Hayes, 2022). To examine the moderating effects of children’s learning behaviors on the relationship between the home digital environment and children’s digital literacy, PROCESS Model 1 was employed. In this model, home digital resources was entered as the independent variable (X), children’s digital literacy (operational or cultural) as the dependent variable (Y), and each learning behavior (competence motivation, attention/persistence, and learning strategy) was entered as a moderator (W) in separate analyses. The significance of interaction effects was tested using a bootstrapping method with 5,000 resamples, and 95% bias-corrected confidence intervals (CIs) were calculated. An interaction effect was considered statistically significant if the CI did not include zero. In addition, the Johnson–Neyman technique was used to identify the regions of significance across the full range of the moderator.

The article "Beyond devices: preschoolers’ learning behaviors as moderators of the link between home digital resources and their digital literacy" was published in 2025. Journal: Front Psychol.

## 4 Results

### 4.1 Descriptive statistics and correlations among the variables

Descriptive statistics and correlations among the key variables are summarized in Table 2.

**Table 2:** Descriptive statistics and correlations among study variables.

Variables	1	2	3	4	5	6
1. Home Digital Resources	1					
2. Competence Motivation	−0.004	1				
3. Attention/Persistence	−0.035	−0.169**	1			
4. Learning Strategy	−0.146**	0.309**	−0.145**	1		
5. Operational Digital Literacy	0.440**	0.082	−0.099*	−0.025	1	
6. Cultural Digital Literacy	0.359**	0.127**	0.112*	−0.132**	0.480**	1
M	0.45	2.49	1.40	2.45	2.26	1.33
SD	0.25	0.34	0.42	0.37	0.50	0.41
Skewness	0.02	−0.61	1.16	−0.62	−0.39	1.72
Kurtosis	−0.68	0.34	1.03	0.29	−0.66	2.94

*p < 0.05, **p < 0.01, ***p < 0.001.

Children had access to about half of the assessed digital devices and tools at home, indicating moderate availability of digital resources in their environments. On average, children showed high levels of competence motivation and learning strategy use, while their ability to sustain attention and persist was relatively lower. This variation in learning behaviors suggests individual differences in how children approach learning tasks.

In terms of digital literacy outcomes, children demonstrated moderate proficiency in operational skills, such as manipulating devices and navigating digital functions. However, cultural digital literacy—which includes creative and interpretive uses of digital media—was generally lower, with some children scoring at the upper limit of the scale, suggesting a potential ceiling effect.

Correlation analyses showed that greater access to digital resources was positively associated with both operational and cultural digital literacy. Children with higher competence motivation and better learning strategy tended to have higher digital literacy scores. Interestingly, learning strategy was negatively associated with cultural digital literacy, implying that children who relied less on structured learning approaches may have engaged more flexibly in digital play. Attention and persistence showed a weak, mixed relationship with literacy outcomes.

The article "Beyond devices: preschoolers’ learning behaviors as moderators of the link between home digital resources and their digital literacy" was published in 2025. Journal: Front Psychol.

These findings provide preliminary support for the idea that both home digital environments and individual learning traits contribute to variations in young children’s digital literacy.

### 4.2 Moderation effects of learning behaviors on the relationship between home digital resources and operational digital literacy

A summary of the interaction effects between home digital resources and each learning behavior on children’s digital literacy is presented in Table 3. In the case of operational digital literacy, the positive effect of home digital resources was found to be stronger for children with higher levels of competence motivation. This means that children who are more intrinsically driven to master tasks and explore tend to benefit more from access to digital resources at home. Even when digital access is similar, those who show stronger motivation are more likely to use digital devices in ways that support skill development—such as navigating apps, adjusting settings, or exploring interactive features. In contrast, children with lower levels of motivation still gained from digital resources, but the benefits were relatively modest. The Johnson–Neyman technique further revealed that the effect of digital access became statistically significant when competence motivation exceeded 1.6935, which included approximately 98% of the sample, suggesting that the moderation effect of competence motivation applied to nearly the entire sample.

**Table 3:** Summary of moderation analyses.

Model	Moderator	Outcome	Interaction (b)	SE	*t*	*p*
1	Competence/ Motivation	Operational DL	0.6028	0.2135	2.82	0.0049
2	Attention/ Persistence	Operational DL	0.0012	0.1775	0.007	0.9947
3	Learning Strategy	Operational DL	0.4069	3.2472	2.01	0.0455
4	Competence	Cultural DL	0.3939	0.1827	2.16	0.0315
5	Attention/ Persistence	Cultural DL	0.0570	0.1514	0.38	0.7069
6	Learning Strategy	Cultural DL	−0.4185	0.1743	−2.40	0.0167

DL, Digital Literacy.

For attention/persistence, no significant interaction was found. This suggests that the degree to which children can focus or persist in tasks did not alter the effect of home digital resources on their operational digital literacy. Regardless of children’s attention spans or persistence levels, the benefit of digital access remained consistent, without evidence of amplification or reduction based on this trait.

In contrast, learning strategy significantly moderated the relationship between home digital resources and operational digital literacy. Children who actively use goal-oriented strategy—such as planning, monitoring, or seeking help—appeared to benefit more from digital tools available at home. Even when digital access was similar, children with higher use of learning strategiy were more likely to engage with digital content in ways that fostered skill development.

The article "Beyond devices: preschoolers’ learning behaviors as moderators of the link between home digital resources and their digital literacy" was published in 2025. Journal: Front Psychol.

The Johnson–Neyman technique identified 1.4204 as the threshold above which the moderating effect of learning strategy became statistically significant, a level that included approximately 99% of the sample. It indicated that the moderation effect of learning strategy was present for nearly the entire sample, suggesting that this is a broadly applicable finding across children with diverse levels of strategy use. These findings suggest that the home digital resources alone is not enough; how children approach learning plays a crucial role in shaping the developmental impact of digital resources. These interaction patterns are further illustrated in Figure 2, which shows how the strength of the relationship between home digital resources and operational digital literacy varies depending on levels of learning behaviors.

**Figure 2:** Interaction effects illustrating the moderation of learning behaviors on the relationship between home digital resources and operational digital literacy.

### 4.3 Moderation effects of learning behaviors on the relationship between home digital resources and cultural digital literacy

For competence motivation, a significant interaction was found in relation to cultural digital literacy. This suggests that the benefits of home digital resources on children’s ability to creatively and interpretively engage with digital content were stronger among children with higher intrinsic motivation. In contrast, children with lower levels of competence motivation also benefited, but to a lesser degree. This pattern implies that motivational dispositions not only drive engagement but also enhance the developmental return from environmental inputs like digital access. The Johnson–Neyman analysis identified a threshold of competence motivation. This threshold covered approximately 97% of the sample, indicating that the moderation effect is relevant for nearly all children with average or higher levels of motivation.

In the case of attention/persistence, the interaction effect on cultural digital literacy was not statistically significant. This suggests that regardless of how well children are able to focus or persist in tasks, the positive association between home digital resources and their cultural digital literacy remained stable.

In the case of learning strategy, a significant negative interaction on cultural digital literacy was found. This suggests that the positive contribution of digital access to children’s cultural digital literacy was stronger among those with lower use of structured learning strategy. In contrast, children who frequently employ structured approaches to learning appeared to benefit less from home digital resources in terms of cultural expression, symbolic engagement, and creative digital play (Figure 3).

The article "Beyond devices: preschoolers’ learning behaviors as moderators of the link between home digital resources and their digital literacy" was published in 2025. Journal: Front Psychol.

**Figure 3:** Interaction effects illustrating the moderation of learning behaviors on the relationship between home digital resources and cultural digital literacy.

This pattern may reflect a compensatory effect of digital exposure: children who are less likely to use goal-directed learning strategy may engage more freely and imaginatively with digital content when provided with access, thereby showing greater gains in cultural digital literacy. Conversely, children with high learning strategy use may already demonstrate structured engagement, leading to a ceiling effect in the contribution of digital access. The Johnson–Neyman analysis did not identify a specific threshold within the observed range. It meant this moderation pattern held across the full range of learning strategy scores, suggesting that the interaction effect was consistent throughout the sample.

Overall, those results implies that digital access alone is not enough; how children approach learning within these environments plays a key role. These findings underscore the importance of considering both structural affordances and child-level learning dispositions in shaping digital literacy development. The interplay between access and approach suggests that tailored support strategy may be needed to optimize digital learning for diverse learners.

## 5 Discussion

The results of this study reveal that preschoolers’ learning behaviors significantly moderated the relationship between home digital resources and preschooler’s digital literacy. By examining each learning behavior subdomain individually—competence motivation, attention/persistence, and learning strategy—this study provides a more nuanced understanding of how each trait uniquely contributes to or constrains children’s acquisition of procedural digital literacy. However, these moderating effects differed by domain: while all three traits generally supported the development of operational digital literacy, their influence on cultural digital literacy was less uniform or even counterproductive in certain contexts. This contrast highlights the importance of domain-specific interventions that align with the cognitive and emotional demands of each digital literacy type.

### 5.1 Moderation effect on operational digital literacy

For operational digital literacy, the results indicated that all three learning behavior traits—competence motivation, attention/persistence, and learning strategy—moderated the relationship between home digital resources and operational digital literacy, though with varying strengths. One of the key findings of this study is that children’s learning behaviors significantly shape how home digital accesses translates into operational digital literacy. Not all children benefit equally from digital resources; rather, those with higher competence motivation, sustained attention, and strategic learning habits are more likely to transform access into meaningful procedural skills.

The article "Beyond devices: preschoolers’ learning behaviors as moderators of the link between home digital resources and their digital literacy" was published in 2025. Journal: Front Psychol.

Among them, competence motivation showed the strongest and most consistent moderating effect. Children with high competence motivation demonstrated a stronger translation of digital access into meaningful outcomes. This subdomain, which reflects a child’s intrinsic drive to master challenges, appears particularly important in the early stages of digital exploration. These children are more likely to initiate interactions with new devices, persist through unfamiliar interfaces, and gradually build their skills over time. The findings suggest that access alone is not sufficient; rather, a child’s willingness to explore and experiment plays a central role in transforming opportunity into learning. This supports Deci and Ryan (1985)‘s view that motivation and autonomy are key engines of development, particularly in self-directed digital environments. Although prior studies (e.g., Razza et al., 2015) emphasized that attentional control plays a critical role in technology-mediated learning, the current study did not find a significant moderating effect of attention/persistence on the relationship between home digital resources and operational digital literacy. This finding indicates that the benefits of home digital resources for children’s procedural digital skills are consistent across different levels of attentional control. In other words, whether children display high or low levels of attention and persistence, access to digital tools contributed similarly to their operational digital literacy. This contrasts with more recent evidence showing that touchscreen-based activities can scaffold preschoolers’ emerging digital literacy when supported by teachers (Neumann, 2022). One possible explanation is that operational skills—such as navigating interfaces, using functions, and following basic procedures—may rely more on repeated exposure and practice than on sustained attention. These results suggest that while attentional control may facilitate deeper or more efficient learning in some contexts, its role as a moderator may be less relevant when children are acquiring foundational operational digital skills. Children with well-developed learning strategy—such as planning, goal-setting, and problem-solving—also showed stronger operational digital literacy when digital resources were available. Strategic use was particularly relevant for navigating menus, adjusting settings, or applying known functions across different tools. However, some limitations emerged: children who relied too heavily on structure may have found it difficult to adapt in open-ended environments that prioritize exploration over task completion. Even so, goal-directed behavior generally strengthened the benefits of digital access. These findings suggest that providing digital tasks with clear objectives and embedded feedback may be particularly effective for children with high levels of strategic engagement. Taken together, the results indicate that each learning behavior contributes differently to the development of operational digital literacy. Competence motivation encourages exploration, attention/persistence sustain it, and learning strategy helps organize actions into meaningful routines. These findings highlight the importance of differentiated support strategy: effective interventions must move beyond access and consider the individual regulatory traits that shape children’s engagement with digital tools.

The article "Beyond devices: preschoolers’ learning behaviors as moderators of the link between home digital resources and their digital literacy" was published in 2025. Journal: Front Psychol.

These results underscore a need for differentiated pedagogical responses. Increasing digital access alone is insufficient. Educators and caregivers should scaffold not only digital skills, but also internal learning traits that enable sustained, autonomous, and adaptable engagement. For example, structured tasks with embedded feedback may support strategic learners, while open-ended challenges can nurture intrinsic motivation.

At the same time, this study raises questions about the fit between structured learning traits and exploratory digital contexts. For some children, an over-reliance on structure may hinder adaptive learning in nonlinear environments. Thus, future interventions should consider how regulatory traits interact with task demands, and avoid one-size-fits-all approaches to digital literacy.

### 5.2 Moderation effect on cultural digital literacy

The moderating effects of learning behaviors on cultural digital literacy were more complex and less consistent than those observed for operational literacy. While competence motivation remained a meaningful influence, attention/persistence and learning strategy appeared less aligned with the developmental demands of this domain. This contrast underscores the importance of distinguishing between types of digital engagement, and recognizing that different forms of literacy may rely on different strengths. Children with strong competence motivation were more likely to engage deeply with symbolic digital content—such as digital storytelling, video narration, or role-play within apps. These forms of engagement often require open-ended exploration, creative thinking, and emotional involvement. Competence motivation may provide the internal drive necessary to persist in such unstructured digital spaces, even in the absence of clearly defined goals. This supports previous findings that intrinsic interest fuels symbolic and creative expression (Cao et al., 2024; Li, 2025; Marsh, 2016; Renninger and Hidi, 2022). Recent work also highlights that digital storytelling and multimedia creation can effectively foster symbolic engagement and creativity in early childhood (Metin et al., 2025). In contrast, attention/persistence did not significantly moderate cultural digital literacy. One possible explanation is that this subdomain is more effective in structured contexts where sustained effort toward a clear outcome is required. Cultural digital tasks—such as imaginative storytelling or artistic exploration—thrive on spontaneity and playfulness rather than continuous focus on a fixed goal. In fact, children who are highly persistent may unintentionally constrain their engagement by trying to impose structure where none is needed. Similarly, learning strategy showed limited or even negative moderation effects on cultural digital literacy. Tasks that involve symbolic play or narrative creation often call for emotional expression and flexibility, which may not align well with a structured, goal-oriented mindset. Children who depend on strategic approaches may seek predefined outcomes and, as a result, engage less fully with open-ended tasks (Ollonen and Kangas, 2025). Systematic reviews also indicate that early digital literacy is closely linked to higher-order cognitive and creative skills, suggesting that cultural digital literacy requires developmental and contextual support (Karnita et al., 2025). Highly structured learners may experience frustration or disengagement in environments that emphasize creativity and interpretation over clear performance criteria. This may be amplified in cultural contexts, such as Korea, where structured performance and adult-led learning are frequently emphasized in preschool settings (Chung et al., 2025). In this light, the negative moderation effect seems unlikely to reflect a statistical ceiling. Instead, it may suggest a broader structural limitation—or what could be considered a floor effect—where children, regardless of their strengths, have limited opportunities to engage with emotionally rich and symbolically meaningful digital experiences. Even children with high levels of strategic engagement may not fully benefit from digital access if their experience is confined to performance-oriented or consumption-based applications. In some cases, highly structured environments may actually disrupt the way they prefer to learn. These findings suggest that the relatively low levels of cultural digital literacy observed in this study may reflect not a lack of ability, but rather a lack of exposure to open-ended, emotionally engaging digital environments.

The article "Beyond devices: preschoolers’ learning behaviors as moderators of the link between home digital resources and their digital literacy" was published in 2025. Journal: Front Psychol.

## 6 Implications

This study underscores that supporting young children’s digital literacy development involves more than simply providing access to digital devices. Meaningful engagement emerges when digital experiences are developmentally appropriate, emotionally resonant, and embedded in relational contexts. While operational digital literacy is often associated with procedural fluency—such as tapping, swiping, and navigating—it is most effectively fostered through repeated hands-on experiences coupled with sensitive adult guidance. Young children benefit from environments that allow them to explore, make mistakes, and try again, particularly when adults provide encouragement rather than control. Parents and educators can facilitate this process by offering digital tools that promote curiosity, problem-solving, and persistence, while responding supportively to children’s efforts. Step-by-step scaffolding may be important initially, but gradually withdrawing adult intervention supports mastery. Selecting digital resources that offer clear feedback, progress cues, and opportunities for self-direction can further enrich children’s learning.

In contrast, cultural digital literacy, which includes symbolic thinking, narrative expression, and socio-emotional communication, requires a different pedagogical approach. This domain flourishes not through structured routines, but through open-ended, imaginative, and emotionally grounded play. Children benefit most when adults engage not as instructors but as co-players—listening, responding, and participating in children’s digital narratives. In such contexts, emotional responsiveness is often more impactful than explicit instruction. To promote cultural digital literacy, caregivers and educators may intentionally integrate digital storytelling, creative drawing tools, multimedia creation, and avatar-based role-play into children’s everyday routines. This aligns with recent findings that digital media practices, such as gamified and collaborative storytelling, can strengthen socio-emotional communication and cultural digital literacy (Li, 2025). These activities are not peripheral but central to how young children construct meaning and communicate in digital spaces. Supporting this kind of engagement involves not only providing tools but also respecting children’s agency, imagination, and expressive voices.

The article "Beyond devices: preschoolers’ learning behaviors as moderators of the link between home digital resources and their digital literacy" was published in 2025. Journal: Front Psychol.

For families, practical support tools such as a “Home Digital Literacy Toolkit” could offer accessible guidance for co-using digital media, identifying developmentally appropriate apps, and encouraging creativity through daily digital routines. Such resources can help parents scaffold both procedural fluency and cultural expression in ways that honor children as active meaning-makers rather than passive users.

This highlights the need for early childhood programs and parenting interventions to prioritize child-led digital contexts that encourage creativity and perspective-taking. Initiatives such as child-directed video production or collaborative story apps can not only enhance digital literacy but also strengthen children’s identity, agency, and relational skills in digital contexts.

Finally, although this study focused on South Korean preschoolers, the findings may resonate in other cultural settings. Future research should examine how parenting styles, cultural values, and levels of digital access interact to shape young children’s learning behaviors and literacy development. Comparative research may uncover both universal mechanisms and culturally specific patterns, helping to build more inclusive and emotionally attuned digital learning environments for children worldwide.

## 7 Limitations, future direction

Several limitations should be acknowledged. The reliance on maternal reports may introduce bias, especially regarding children’s behaviors and digital use. The cross-sectional design limits causal inference; future research should adopt longitudinal or experimental designs to clarify developmental trajectories. Additionally, the focus on mothers excludes the potential role of fathers or teachers in digital mediation. Finally, although this study accounted for internal traits and home environments, broader ecological contexts such as peer influence and institutional practices should also be explored.

Building on these limitations, future research should aim to capture a more comprehensive ecological perspective by incorporating multiple informants (e.g., fathers, teachers, or peers) and observational data to validate children’s learning behaviors and digital engagement. Longitudinal studies are particularly needed to examine how the effects of learning behaviors unfold over time and whether certain traits become more or less influential as children grow and their digital experiences diversify. Additionally, exploring cultural variation in techno-subsystem structures and parenting styles may help to identify universal versus context-specific patterns in digital literacy development. Finally, while this study focused on operational and cultural digital literacy, future work should investigate how learning behaviors relate to the emergence of critical digital literacy in middle childhood and beyond. Systematic reviews have emphasized that digital literacy development in early childhood is increasingly linked to higher-order cognitive and creative skills (Karnita et al., 2025), suggesting the need to trace developmental transitions over time. Future research should further examine how home and technological contexts provide opportunities for symbolic and creative digital engagement. Emerging platforms such as virtual or augmented reality (Navarro and Tudge, 2022) also merit investigation as potential contexts for developing cultural digital literacy.

The article "Beyond devices: preschoolers’ learning behaviors as moderators of the link between home digital resources and their digital literacy" was published in 2025. Journal: Front Psychol.

## 8 Conclusion

This study offers new insight into how young children’s digital literacy develops, emphasizing the interaction between their internal learning traits and the digital opportunities present at home. By applying Bronfenbrenner’s bioecological model and distinguishing between operational and cultural literacy, this work highlights that children’s learning behaviors—especially competence motivation—play a crucial moderating role. As digital technology becomes increasingly woven into early childhood, it is essential to consider not just what tools are available, but how children experience them. Moving forward, future studies should consider more diverse social agents (like peers and teachers), track developmental changes over time, and expand to include critical digital literacy as children grow into more autonomous digital participants.

## Data Availability

The datasets presented in this article are not readily available because data from this study cannot be distributed, as participant consent for public sharing was not obtained. Requests to access the datasets should be directed to moonyk@dju.kr.
